# Anticancer Activities of Protopanaxadiol- and Protopanaxatriol-Type Ginsenosides and Their Metabolites

**DOI:** 10.1155/2016/5738694

**Published:** 2016-06-30

**Authors:** Xiao-Jia Chen, Xiao-Jing Zhang, Yan-Mei Shui, Jian-Bo Wan, Jian-Li Gao

**Affiliations:** ^1^State Key Laboratory of Quality Research in Chinese Medicine, Institute of Chinese Medical Sciences, University of Macau, Macau; ^2^Zhejiang Chinese Medical University, Hangzhou, Zhejiang 310053, China

## Abstract

Recently, most anticancer drugs are derived from natural resources such as marine, microbial, and botanical sources, but the low success rates of chemotherapies and the development of multidrug resistance emphasize the importance of discovering new compounds that are both safe and effective against cancer. Ginseng types, including Asian ginseng, American ginseng, and notoginseng, have been used traditionally to treat various diseases, due to their immunomodulatory, neuroprotective, antioxidative, and antitumor activities. Accumulating reports have shown that ginsenosides, the major active component of ginseng, were helpful for tumor treatment. 20(*S*)-Protopanaxadiol (PDS) and 20(*S*)-protopanaxatriol saponins (PTS) are two characteristic types of triterpenoid saponins in ginsenosides. PTS holds capacity to interfere with crucial metabolism, while PDS could affect cell cycle distribution and prodeath signaling. This review aims at providing an overview of PTS and PDS, as well as their metabolites, regarding their different anticancer effects with the proposal that these compounds might be potent additions to the current chemotherapeutic strategy against cancer.

## 1. Introduction

Cancer is a group of diseases characterized by evading growth suppressors, activating invasion and metastasis, avoiding immune destruction, and deregulating cellular anabolism and metabolism. In 2015, a total of 1,658,370 new cancer cases and 589,430 cancer deaths were projected to occur in the United States [1]. In China, the estimates of new cancer incident cases and cancer deaths were 3,372,175 and 2,113,048, respectively [2]. However, chemotherapy always suffered from increasing multidrug resistance. Thus, identifying more chemicals extracted from herbal medicines is an essential step in advancing cancer treatment. Nowadays, many herbs, typically ginseng and notoginseng, have been used in clinical practice to treat advanced cancer in eastern countries, and researchers pay more and more attention to the potential therapeutic effects of those herbs. Therefore, it is very important to understand the bioactive effects and mechanism of the main ingredients and absorbed metabolites of these herbs.

Asian ginseng, American ginseng, and notoginseng, the roots and rhizome of* Panax ginseng* C. A. Meyer,* Panax quinquefolius* L., and* Panax notoginseng* (Burk.) F. H. Chen, belong to genus* Panax* of the family Araliaceae. These herbs have long been used for preventive and therapeutic purposes for thousands of years in Asian and North American countries.* Ben Cao Gang Mu* recorded that Asian ginseng was usually used as a tonic, sedative, life-prolonging, or gastrointestinal regulation drug to treat fatigue, blood deficiency, insomnia, and impotence [3]. American ginseng was first recorded in* Ben Cao Cong Xin* in 1757 and was used for relieving internal heat, cough, bloody phlegm, dysphoria and tiredness, and dry and thirsty mouth and throat. Notoginseng, another herb belonging to the genus* Panax*, is well known for treatment of blood disorders. Notoginseng is usually available in two different forms: the raw and steamed (processed) forms. The raw notoginseng has been traditionally used for its hemostatic and cardiovascular effects to arrest internal and external bleeding, reduce swelling and pain, and remove blood stasis and promote blood circulation [4]. Unlike raw notoginseng, the steamed form has been widely accepted to be a tonic to “nourish” the blood and to increase blood cells in anemic conditions [5].

Modern studies showed that Asian ginseng, American ginseng, and notoginseng exhibited various significant pharmacological effects, and the anticancer activities of ginseng types have been extensively investigated based on the functional capacity of inhibiting cancer cell growth, inducing angiogenesis, delaying invasion and metastasis, and regulating tumor-related immune suppression by their active ingredients, ginsenosides and their metabolites [6, 7]. PDS (20(*S*)-protopanaxadiol (PPD) saponins) and PTS (20(*S*)-protopanaxatriol (PPT) saponins) and their metabolites are the major anticancer active components of the most popular* Panax* herbs. Notably, ginsenoside Rg3 was produced as an antiangiogenic drug in China. In this review, we summarize and compare the regulatory effects of different ginsenosides and their metabolites on the development of cancer, and the corresponding mechanisms have also been discussed.

## 2. Chemical Structures and Metabolism of PDS and PTS

Saponins and sapogenins of ginseng types (also named ginsenosides) are the major bioactive constituents which were possibly responsible for the comparable and distinct pharmacological activities in the three* Panax* herbs [8]. All of the total ginsenosides extracts of these three herbs are chemical mixtures containing a group of triterpene glycosides with similar ingredients and structure, which have been shown to possess anticancer, anti-inflammatory, and neuroprotective activities and promote blood circulation to treat cardiocerebrovascular diseases [9]. Nowadays, more than sixty individual saponins were isolated from these three* Panax* herbs. They are classified into two main groups according to the different aglycone, namely, PDS, such as ginsenoside Rb1, and PTS, such as ginsenoside Rg1. The two types of triterpenoid saponins showed diverse or even antagonistic pharmacological activities [10]. Cumulated researches elucidated that the content of total saponins in notoginseng is higher than those in Asian ginseng [11], while ginsenosides Rb1, Re, and Rg1 are enriched in American ginseng, and ginsenosides Rf and Rb2 are enriched in Asian ginseng [12].

It is noteworthy that PDS and PTS are not easily absorbed by the body through the intestines due to their hydrophilicity [13]. Little amount of PDS could be absorbed in the gastrointestinal tract following oral intake. Therefore, these constituents inevitably come into contact with and are metabolized by microflora in the alimentary tract. As shown in Figure 1, upon oral consumption, ginsenosides are partly transformed into the PPD and PPT through a series of deglycosylation procedures by acid hydrolysis and intestinal bacterial actions [14]. All of the metabolites, such as compound K (CK), PPD, and PPT, are nonpolar compared to the parental components ginsenosides, which could be easily absorbed in the gastrointestinal tract and express biological actions [15]. The ability of PPD to be absorbed after oral administration had been demonstrated through pharmacokinetic studies. It was shown that PPD accumulated largely in the stomach (44%) and small in the intestine (32%) and was also present in the brain (0.01%) [16].

Many reports reveal that the metabolites were assessed as more potent bioactive ingredients than the natural ones. It is validated that PPD, a stable deglycosylated PDS metabolic derivative that could be formulated for oral gavage, exerted antineoplastic actions, which were more effective than its prototype [17]. A good example is the improved anti-androgen-independent prostate cancer activity exerted by the intestinal bacterial metabolites compared to natural occurring ginsenosides, through decreasing survival rate, inhibiting proliferation, inducing apoptosis, and leading to cell cycle arrest in PC-3 cells [18]. The increase of lipotropy and decrease of C-6 steric hindrance, which were caused by deglycosylation by intestinal bacteria, might be the reason for the higher activity of metabolites.

## 3. Anticancer Effects of Ginsenosides

Preclinical and clinical researches demonstrated that ginsenosides have cancer preventing activities to various tumors, including gastric carcinoma, breast cancer, liver cancer, ovarian cancer, colon cancer, melanoma, and leukemia [19]. Extensive phytochemical and pharmacological studies on ginseng and notoginseng proved that the PDS and PTS are the main anticancer compositions and that the activities of PDS were more powerful than those of PTS [15, 20, 21]. In general, the anticancer effects of total ginsenoside from Asian ginseng and American ginseng, but not notoginseng, are widely reported; meanwhile, lots of publications indicated the anticancer effects of many pure ginsenosides, such as ginsenosides Rg3 and Rh2, isolated from all of the three ginseng types. In view of the results reported by Lee et al. [20] and Jin et al. [21], the relative nonpolar and PDS class ginsenosides exhibited more cytotoxicity on breast cancer cells and efficient cellular uptake on MCF-7 and MCF-7/MX cells compared with the relative polar and PTS class compounds. Shim et al. [15] suggested that the PDS and ginsenosides Rd, Rg3, Rk1, Rg5, and Rh2 showed potent or moderate inhibitory activities on inducing apoptosis of cancer cells through activating the caspase-3 pathway, whereas the PTS and ginsenosides Rf, Rg1, Re, Rh1, and Rg2 did not exhibit any inhibitory activity.

The structure-activity relationships indicated that both glycosylation at C-3-OH and nonoxidation at C-6 on ginsenosides might be important for the inhibition of the chymotrypsin-like activity of the 20S proteasome which plays an important role in selective protein degradation and regulates cellular events in anticancer process. On the other hand, several results indicate compound with less polar chemical structures possesses higher cytotoxic activity towards cancer cells. The ginsenosides with two molecules of glucose linked to C-3-OH have a less potent inhibitory activity than those with one molecule; for example, Rh2 (one glucose at C-3) showed more potent pharmacological activities than Rg3 (two types of glucose at C-3) [7]. From this perspective, cytotoxic potencies of the hydrolysates of PDS and PTS, especially PPD and CK (the hydrolysate of PPD-type ginsenoside fractions), are much stronger than the original ginsenosides.

It appears that CK, Rh2, Rg3, PPD, and PPT are possibly responsible for the enhanced anticancer activity of ginseng. In fact, processing of herbs could change the chromatographic and pharmacological profiles of notoginseng and cause an increase of PDS and its hydrolysates, including ginsenosides Rh2, Rk1, Rk3, and Rg3, which might contribute to the greater antiproliferative effects against liver cancer cells, SNU449, SNU182, and HepG2 of steamed notoginseng than its raw form [22]. In another case, Lin et al. [23] attested that, after lactic acid bacteria fermentation, antihepatocarcinoma activity of notoginseng was improved, along with the fact that notoginsenoside R1 and ginsenosides Rg1, Rb1, Rd, and Rh4 were decreased, while ginsenosides Rh1 and Rg3 were increased during fermentation. Additionally, after it is orally taken, PTS would be inevitably deglycosylated by intestinal bacteria. For instance, biotransformation of ginsenoside Rg1 by the fungus* Absidia coerulea* AS3.2462 yielded five metabolites. Three of them exhibited moderate reversal activity towards A549/taxol MDR tumor cells* in vitro* [24]. The therapeutic targets of ginsenosides on cancer were summarized in Figure 2.

### 3.1. Inhibiting Cancer Cell Growth

Extensive experiment data indicates that ginsenosides could inhibit tumor growth by inhibiting cancer cell proliferation, which can be related with inducing apoptosis and autophage of cancer cells, inhibiting proliferative signaling pathways, or regulating the activity of tumor suppressors. For instance, ginsenoside Rh1 showed great estrogenic effect in human breast carcinoma MCF-7 cells [25]. The synthesized monoester of ginsenoside Rh1 showed moderate effects on murine H22 hepatoma cells [26]. Yang et al. [27] suggested that ginsenoside Rd could serve as a lead to develop novel chemotherapeutic or chemopreventive agents against human cervical cancer.

#### 3.1.1. Inducing Apoptosis and Autophage of Cancer Cells

*(1) PPD*. Nowadays, PPD has been well characterized to possess the pleiotropic anticarcinogenesis capabilities in many cancer cell lines, including A172, A549, B16, Caco-2, Ehrlich ascites cells L1210, H1299, H358, H838, HCT-116, HCT-8, HeLa, HepG2, HPAC, Int-407, Jurkat, LNCaP, MCF-7, MDA-MB-468, Me180, Molt-4, Panc-1, P388, PC3, Raji, SK-HEP-1, SW-480, T98G, and THP-1. PPD could induce different forms of programmed cell death, including typical apoptosis and autophagy through both caspase-dependent and caspase-independent mechanisms, which could be testified in models of two human glioma cell lines, SF188 and U87MG. For the SF188 cells, PPD activated caspase-3, caspase-7, caspase-8, and caspase-9 and induced rapid apoptosis. Interestingly, in U87MG cells PPD induces cell death without activating any caspases, but with promoting the dramatic autophagy of cells [28]. Additionally, PPD induced the intrinsic and extrinsic apoptotic pathways, activated death receptor 5 and caspase-3, caspase-8, and caspase-9, and upregulated the mRNA and/or protein levels of endoplasmic reticulum stress-associated molecules in HepG2 cells [29]. The research reported by Popovich and Kitts [30] showed that PPD possessed characteristic effects on the proliferation of human leukemia cells THP-1 and that the presence of sugars in PPD aglycone structures reduced the potency to induce apoptosis. It could also inhibit the growth of acute lymphoblastic leukemia (ALL) cell lines Reh and RS411 cells by stimulating differentiation and inhibiting growth and cell cycle progression of ALL cells without changing cell apoptosis [31].

The analogue of PPD is now also known to be helpful for tumor treatment. 20(*S*)-25-Methoxyl-dammarane-3*β*,12*β*,20-triol (25-OCH_3_-PPD) is a dammarane-type triterpene sapogenin isolated from* P. notoginseng*, which has been regarded as the principal medicinal component of the plant and has shown anticancer effects* in vitro* and* in vivo* with a low toxicity to noncancer cells [32]. Bi et al. [33] added it to LS174, SW620, SW480, and A549 cells and demonstrated that it significantly inhibited cell proliferation and induced apoptosis by modulation on *β*-catenin, a key mediator in the Wnt pathway. Meanwhile, other researchers found that 25-OCH_3_-PPD exhibited activity against human H358 and H838 lung cancer cells and androgen-dependent prostate cancer cells, LNCaP and PC3, through decreasing survival, inhibiting proliferation, and inducing apoptosis and G_1_ cell cycle arrest. This compound also decreased the levels of cell proliferation-associated proteins (MDM2, E2F1, cyclin D1, and cyclin-dependent kinase 2 (CDK2) and CDK4) and increased the activation of proapoptotic proteins (cleaved PARP, cleaved caspase-3, caspase-8, and caspase-9) [32]. Wu et al. [34] detected that 25-OCH_3_-PPD produced a significant inhibitory effect on activated t-HSC/Cl-6 cells based on its regulatory function to increase the level of cellular GSH and cleaved caspase-3, while PPT, Rg3, Rb1, Rb3, Rg1, Rg2, and Re showed little or no cytotoxic effects. Aside from 25-OCH_3_-PPD, 20(*R*)-dammarane-3*β*,12*β*,20,25-tetrol (25-OH-PPD) has abilities to inhibit proliferation, leading to cycle arrest, inducing apoptosis on cancer cells, and inhibiting the growth of xenograft tumors without any host toxicity [35].

*(2) CK*. 20-O-D-Glucopyranosyl-20(*S*)-protopanaxadiol (CK, IH-901, or M1), one of the most important metabolites of PDS by intestinal microorganisms, is drawing increasing attention recently due to its potent inhibitory benefits on cancer, including hepatocarcinoma cells, breast cancer cells, lymphoma cells, and melanoma cells,* in vitro* and* in vivo* (shown in Table 1) [36]. The IC_50_ of CK to inhibit the proliferation was 12.7, 11.4, 8.5, and 9.7 *μ*M for B16-BL6, HepG2, K562, and 95-D cell lines, respectively [37]. Oral administration of CK significantly inhibited the tumor proliferation at the implantation site after intrapulmonary implantation of Lewis lung carcinoma and colon 26-L5 tumor cells in concentration- and time-dependent manners and suppressed the metastasis to meditational lymph nodes, which was primarily due to induce caspase-3-dependent apoptosis [38]. Moreover, the analogue of CK, 3-O-oleoyl CK (OCK), caused 2.6-fold suppression of tumor growth compared with CK on the growth and metastasis of murine B16-F10 melanoma cells in C57BL/6 mice [39].

CK exhibits cytotoxicity largely by inducing apoptosis via generation of reactive oxygen species (ROS), regulating on cell cycle arrest at the G_1_ phase, upregulating Bax, disrupting the mitochondrial membrane potential, activating caspase-3, caspase-8, and caspase-9, inhibiting of telomerase activity, and decreasing cyclooxygenase-2 (COX-2) expression and prostaglandin E_2_ (PGE_2_) levels via an AMP-activated protein kinase- (AMPK-) dependent pathway [40]. The treatment of MDA-MB-231 with CK upregulated COX-2 mRNA and protein and enhanced the production of PGE_2_ [41]. Hu et al. [42] and Cho et al. [43] reported that CK significantly inhibits the viabilities of BGC823, SGC7901, and HL-60 cells in dose- and time-dependent manners mainly through mitochondria-mediated internal pathway. In the HL-60 treatment, this compound still induced a series of intracellular events associated with death receptor-dependent apoptotic pathway [43].

Meanwhile, CK led to G_1_ cell cycle arrest in tumor cells. Exposure to CK for 48 hours led to G_1_ arrest in Hep3B, U937 cells, MDA-MB-231, Hs578T, and MKN28 cells [40, 41, 44]. The CK-mediated G_1_ arrest resulted from an increase in p27^Kip1^ mRNA and protein expression followed by a decrease in CDK2 kinase activity. Saiki [45] proposed that the induction of apoptosis of tumor cells by CK involved the upregulation of the CDK inhibitor p27^Kip1^ as well as the downregulation of c-Myc and cyclin D1 in a time-dependent manner.

In addition to PPD and CK, Rh2 and Rg3 may be also effective preclinical candidate compounds for liver cancer, breast cancer, prostatic cancer, pediatric acute myeloid leukemia and glioblastoma, and so forth (shown in Table 1). X. Wang and Y. Wang indicated that Rh2 significantly prolonged the survival of mice with pediatric leukemia and induced apoptosis of leukemia cells through miR-21-modulated suppression of Bcl-2 [46]. Liu et al. found that Rh2 dose-dependently reduced SCC viability and increased autophagy and reduced *β*-catenin signaling in SCC cells [47].

#### 3.1.2. Inhibiting Proliferative Signaling Pathways

Besides the activities mentioned above, PPD and CK can exert their anticancer effect through direct antiproliferation activation. In fact, our results suggest that the anticancer activity of PPD in colon cancer cells may be mediated through targeting multiple cancer signaling pathways, namely, nuclear factor-kappa B (NF-*κ*B), JNK, and mitogen-activated protein kinase (MAPK)/extracellular signal-regulated kinase (ERK) signaling pathways [48]. Hwang et al. [49] also demonstrated the antiproliferative and proapoptotic effects of an enzymatically fortified ginseng extract on KATO3 cells appear to be associated with the upregulation of Bax, the activation of NF-*κ*B, and the inhibition of mTOR and PKB signals. PPD also downregulates the PI3K/Akt signaling pathway in A549 cells [50]. Yu et al. [51] found that PPD inhibited estrogen-stimulated gene expression and cell proliferation both* in vitro* and* in vivo* through blocking [^3^H]-17-*β*-estradiol- (E_2_-) induced transcriptional activation and inhibiting colony formation of endometrial cancer cells. Kang et al. described the fact that CK induced the activation of c-Jun N-terminal kinase (JNK) and the transcription factor AP-1, a downstream target of JNK [44]. Furthermore, CK induced apoptosis and inhibits fibroblast growth factor receptor 3 (FGFR3) expression and signaling in myeloma cell line KMS-11, suggesting candidacy for the chemoprevention and the treatment of myeloma [52].

CK also depresses several cell proliferation signaling pathways, for example, ERK, Janus activated kinase (JAK) 1/signal transducer and activator of transcription 3 (STAT3), AMPK pathway, and FGFR3 signaling. The treatment of MDA-MB-231 with CK upregulated COX-2 mRNA and protein, enhanced the production of PGE_2_, and induced the sustained activation of ERK [41]. Furthermore, CK inhibited phosphorylation of STAT3 and its upstream activator, JAK1, but not JAK2, downregulated STAT3 target genes bcl-x_L_, bcl-2, survivin, cyclin E, and D1, and enhanced the expression of protein tyrosine phosphatase SHP-1, but not phosphatase and tensin homolog (PTEN) in this treatment [53].

Similar to PPD and CK, other PDS also target in the cancer cell proliferation related signaling pathways. For example, our results strongly suggest that ginsenoside Rg3 diminishes nuclear staining intensity of *β*-catenin; the anticancer activity of Rg3 may be in part caused by blocking the nuclear translocation of *β*-catenin in colon cancer cells [54]. Besides, treatment with ginsenoside Rd dose- and time-dependently inhibited the migration and invasion of human hepatocellular carcinoma HepG2, Hep3B, SNU-398, and SNU-878 cells via blocking MAPK signaling, inhibiting the phosphorylation of ERK and p38 MAPK, inhibiting AP-1 activation [55].

#### 3.1.3. Regulating the Activity of Tumor Suppressors

Tumor suppressor, such as p53, VHL, ING4, Rb, PTEN, p16, p21, APC, DCC, NF1, NF2, WT1, and DR4 death receptor, is a type of genes that protects a cell from one step on the path to cancer [56]. Defects in the tumor suppressor pathway make tumors vulnerable to varieties of stresses, which can be exploited therapeutically. CK inhibits HCT-116, SW-480, and HT-29 cancer cell growth by upregulation of p53/p21, FoxO3a-p27/p15, and Smad3 and downregulation of cdc25A, CDK4/CDK6, and cyclin D1/3 [57]. Similarly, PPD could activate p53 and p21 and downregulate the levels of CDK2, cyclin E and cyclin D1, and PCNA in NIH3T3 cells [58].

As shown in Table 1, several other PDS, such as ginsenosides Rg3, Rh2, Rk1, and Rs3, also demonstrated activation of the activity of p53 and p21 [59]. Rs3 could elevate the protein levels of p53 and p21^WAF1^ and then downregulate the activities of the cyclin-dependent kinases in SK-HEP-1 cells [60]. Sin et al. indicated that Rg3 could induce senescence-like growth arrest by regulating Akt and p53/p21-dependent signaling pathways in human glioma cells [61]. Rg3-mediated phosphorylation of p53 resulted in inhibition of Akt phosphorylation, which in turn reduced MDM2-mediated p53 degradation [62]. Rg3 also has antiproliferative activity against melanoma by decreasing HDAC3 and increasing acetylation of p53 on lysine (k373/k382) both* in vitro* and* in vivo* [63]. Moreover, Rh2 induces apoptosis and paraptosis-like cell death in colorectal cancer cells through activation of p53 [64] and increases the expression level of DR4 death receptor [65]. Guo et al. [66] found that significant increases in Fas expression and caspase-8 activity temporally coincided with an increase in p53 expression in p53-nonmutated HeLa and SK-HEP-1 cells upon Rh2 treatment.

### 3.2. Antiangiogenesis

Tumor-induced angiogenesis (neovascularization) is one of the most important events concerning tumor growth and metastasis [45]. As shown in Tables 1 and 2, PPT, PPD, and several PDS, namely, CK, Rg3, Rh2, Rb1, and F2, presented significantly antiangiogenic effect. Through investigating their antiangiogenic effects in an angiogenesis model of human umbilical vein endothelial cells (HUVECs), Usami et al. [67] found that PPD displayed inhibition on proliferative activity of HUVECs in a dose-dependent manner and had potential as anticancer drug candidates.

Jeong et al. [68] investigated the antiangiogenic activity and relative mechanisms of CK in HUVECs. The outcomes revealed that CK significantly inhibited the proliferation and downregulated phosphorylation of p38 MAPK and AKT in bFGF treated HUVECs. Besides, it inhibited the migration and tube formation, reduced secreted level of vascular endothelial growth factor (VEGF), and increased the secreted level of pigment epithelium-derived factor (PEDF) at noncytotoxic concentrations.* In vivo* experimental results revealed that CK effectively disrupted bFGF-induced neovascularization in the Matrigel plugs excised from mice and inhibited the tumor formation of SGC7901 cells in nude mice [42, 68].

Recently, 20(*S*)-ginsenoside Rg3 was produced as a new anticancer drug in China due to its antiangiogenic effect. Clinical studies show that Rg3, especially in combination with chemotherapy, can reduce chemotherapy side effect and improve life quality and survival rates of patients with non-small cell lung cancer [171], gastric cancer [172], esophageal cancer [173], and so forth. The mechanism might be correlated with antitumor angiogenesis and improving the immune function. The results were confirmed in many animal models, such as C57BL/6 mice bearing Lewis lung tumor model and rabbits inoculated with liver VX2 tumor model. Yu et al. found that Rg3 could suppress the tumor growth and angiogenesis in VX2 transplanted hepatic tumor model in experimental rabbits. The tumor microvessel density (MVD) and the expression of VEGF were significantly lower than those of the control group [174]. Rg3 also enhanced the antiangiogenic of capecitabine in a model of BALB/c mice inoculated with 4T1 breast cancer [175] and inhibited neovascularization and growth of mouse Lewis lung carcinoma with gemcitabine in C57BL/6 mice inoculated with Lewis lung carcinoma [176].

### 3.3. Delaying Invasion and Metastasis

Besides the activities mentioned above, some compounds belong to PDS and PTS also exert other pharmacological effects about anticancer. PDS and its metabolites, including Rb2, Rd, F2, Rh2, Rg3, CK, and PPD, could inhibit the tumor invasion and metastasis. Moreover, PTS (shown in Table 2) and its metabolites, including Rg1, Rh1, and PPT, also affect the tumor invasion and metastasis process. Inhibiting epithelial-mesenchymal transition (EMT) and regulating the expression and activity of cellular adhesive molecules, matrix metalloproteinases (MMPs), and collagenases are involved in the anti-invasion effect of ginsenosides.

The results obtained by Li et al. [73] indicated that PPD significantly inhibited the invasiveness of HT1080 cells* in vitro*, and this action is primarily due to downregulating the expression of MMP-2. Cathcart et al. found that ginsenoside Rd dose- and time-dependently inhibited the migration and invasion of human hepatocellular carcinoma HepG2, Hep3B, SNU-398, and SNU-878 cells via reducing the expression of MMP-1, MMP-2, and MMP-7 [177] and inducing focal adhesion formation and modulating vinculin localization and expression [55].

Other reports indicated that both Rg1 and Rg3 suppress liver cancer cell HepG2 or lung cancer cell A549 migration and invasion* in vitro* by inhibiting the transforming growth factor- (TGF-) *β*1-induced EMT [161, 178]. The anti-invasion effects of Rg3 and Rh2 were proved related with the expression of MMP-13 both in B16F10 mouse melanoma cancer cells and in glioblastoma multiforme cells [179, 180]. 20(*S*)-Rg3 also effectively inhibits EMT in nude mouse xenograft models of ovarian cancer by blocking hypoxia-induced epithelial-mesenchymal transition [92] and limited metastasis and promoted survival by downregulating VEGF overexpression in HCC tumor [181].

### 3.4. Regulating of Tumor-Related Immune Suppression

The evidences support the effect of ginsenosides on overcoming tumor to evade the immune system. Wang et al. [182] reported that CK could inhibit tumor growth by decreasing the expressions of immunosuppression-related gene and suppressing the production of proinflammatory cytokines. Hao et al. found that total ginsenosides from Asian ginseng can promote the growth inhibition and apoptosis of human T lymphocyte Jurkat cells induced by PG human lung carcinoma cells, which may be related to the upregulation of cytokine TGF-*β*1 secretion in PG cells [183]. Zhou et al. [184] have compared the anticancer activity of CK plus cyclophosphamide (CTX) with that of CTX alone. The result exhibited that the combination effect was significantly superior and synergistic, which might due to immunoregulation activity of CK by improving the WBC, interleukin- (IL-) 2, and interferon- (IFN-) *γ* degraded of CTX. Further studies implied that OCK did not directly affect tumor growth* in vitro*, whereas it promoted tumor cell lysis by lymphocytes, particularly nonadherent splenocytes [185].

Dendritic cell (DC) plays a pivotal role in the initiation of T cell-mediated immune responses through influencing T cell differentiation towards the Th1, Th2, or Th17 type and regulating factors related to the direction of the T cell polarization [186]. PPT exerts anticancer bioactivity mainly through its ability to improve immunity on DC-based vaccines [187], and the activity of PPT is stronger than its original ginsenosides form, PTS. Stimulation with 20 *μ*M of PPT increased expression of CD80, CD83, and CD86 and decreased endocytic activity in DCs [188]. As the most important anticancer compound in ginseng, Rg3 also presented inhibition of tumor growth and immunomodulation activities in H22-tumor bearing mice attributed to the improvement of cellular immunity. It could stimulate ConA-induced lymphocyte proliferation and augmentation of Th1-type cytokines IL-2 and INF-*γ* levels in mice [101].

In addition to the above, ginsenosides also improve the immune destruction of organism. Jang et al. [189] indicated that methanol extract of cultured wild ginseng cambial meristematic cells (CMCs) is effective for potentiation of NK cell and anticancer activity. PPT-primed mature DCs displayed enhanced T cells stimulatory capacity in an allogeneic mixed lymphocyte reaction. Mature DCs differentiated with PPT induced the differentiation of naive T cells towards a Th1 response. The production of IFN-*γ* and ^51^Cr release on PPT-primed mature DCs was augmented, while small amounts of IL-4 depending on IL-12 secretion were investigated [188].

### 3.5. Deregulating Cellular Anabolism and Metabolism

More and more evidence indicated that the anticancer effect of ginsenosides is also related with its abilities on regulating abnormal tumor anabolism, metabolism, and glycolysis. Li et al. [190] showed that 20(*S*)-Rg3 could inhibit Warburg effect through STAT3/HK2 pathways, and 20(*S*)-Rg3 decreased metabolic enzymes in glycolysis including PKM2, HK2, GLUT1, and LDH, but the mechanism still needed further study. Aglycone of Rh4 inhibits melanin synthesis in B16 melanoma cells via the protein kinase A pathway [191]. Investigations indicated that Rh4 significantly reduced the cyclic AMP (cAMP) level and downregulated microphthalmia-associated transcription factor and tyrosinase in B16 melanoma cells. Otherwise, Rg1 has been shown to bind to the glucocorticoid receptor (GR), leading to the downregulation of GR expression and the induction of GR-mediated transcription synergistically with cAMP in FTO2B rat hepatoma cells [192].

As a kind of aldose reductase inhibitor, Rh2 induced AMPK and p38 MAPK activation and thus determined the apoptotic sensitivity of cancer cells [111]. Rg3 and its metabolite CK also impact on the cancer-related metabolism pathways like AMPK. Yuan et al. found that Rg3-induced apoptosis in HT-29 colon cancer cells is associated with AMPK signaling pathway [193]. CK-mediated cell death of HT-29 colon cancer cells is regulated by calcium/calmodulin-dependent protein kinase- (CAMK-) IV/AMPK pathways [126] and CK induced apoptosis by modulating AMPK-COX-2 signaling in MCF-7 human breast cancer cells [40].

### 3.6. Inhibiting Tumor-Prompting Inflammation

Tumor promotion often accompanies an elevated ornithine decarboxylase (ODC) activity, acute inflammation, and induction of COX-2 activity, and the eukaryotic transcription factor NF-*κ*B has been involved in intracellular signaling pathways associated with inflammation and carcinogenesis [194]. CK has been reported to possess anti-inflammatory effects by inhibiting 12-O-tetradecanoylphorbol-13-acetate- (TPA-) induced COX-2 expression. Lee et al. [195] showed that topical application of CK onto shaven backs of female ICR mice led to the inhibition of TPA-induced expression of COX-2 and production of PGE_2_. CK pretreatment inhibited TPA-induced epidermal NF-*κ*B DNA binding in mouse skin, which appeared to be mediated by blocking phosphorylation and subsequent degradation of I*κ*B*α*. The regulatory effect on COX-2 and NF-*κ*B has also been found in Rg3-pretreated mouse skin stimulated by TPA [104].

### 3.7. Depressing Carcinogenesis

Eliminating and reducing risk factors of carcinogenesis are considered a critical step to tumor prevention and control. Korean investigators carried out extensive long-term anticarcinogenicity experiments with 2000 newborn mice stimulated by several chemical carcinogens and suggested that traditional Chinese medicine ginseng holds a potential anticancer effect [196]. There was a 22% decrease (*p* < 0.05) in the incidence of urethane induced lung adenoma by the use of red ginseng extract. Yun and colleagues indicated that red ginseng extract showed inhibition of lung tumor incidence, while fresh ginseng did not [196]. Another research from Yun's group also demonstrated that the anticarcinogenicity of ginseng was more prominent in aged or heat treated extracts of ginseng and red ginseng made by steaming. Moreover, ginsenosides Rg3, Rg5, and Rh2 were found to be active anticarcinogenic compounds [103].

The report by Keum and colleagues suggested that Rg3 also inhibits the tumor promotion. Pretreatment of dorsal skins of female ICR mice with Rg3 significantly inhibited TPA-induced ornithine decarboxylase activity and 7,12-dimethylbenz[a]anthracene-initiated papilloma formation. Rg3 pretreatment also abrogated the expression of COX-2 in TPA-stimulated mouse skin possibly through downregulation of NF-*κ*B and AP-1 transcription factors [104]. Furthermore, Rb2 prevents human cancers by downregulation of gap junctional intercellular communication by TPA and hydrogen peroxide in WB-F344 rat liver epithelial cells [142]. CK could prevent tumorigenesis of aberrant crypts in C57BL:6 mice colonized with ginseng-hydrolyzing bacteria [197].

Phase 2 detoxification enzymes protect against carcinogenesis and oxidative stress. Lee et al. [198] illustrated that PPD induced the activity of phase 2 detoxification enzymes. Ginseng extracts and components (such as PPD and PPT) were assayed for inducer activity of NQO1 (quinone reductase), a phase 2 enzyme, in Hepa1c1c7 cells. Wang et al. [140] suggested that the chemopreventive effect of* Panax ginseng* may be also due, in part, to ginsenosides Rg1 and Rb1's ability to compete with aryl hydrocarbons for both the aryl hydrocarbon receptor and CYP1A1 in HepG2 cell.

### 3.8. Synergy with Chemotherapy

It is suggested that the combination of ginsenoside or notoginsenoside with chemotherapy drugs acts synergistically to produce therapeutic effects greater than those that can be achieved with single use. With the aim of increasing the activities and decreasing the side effects, the adjuvant potentials of saponins had been screened. Combining 25-OCH_3_-PPD with conventional chemotherapeutic agents or radiation led to potent anticancer effects. The tumor regression was almost complete following administration of 25-OCH_3_-PPD and taxotere/gemcitabine [35]. Researchers had also hypothesized that the potential therapeutic efficacy of PTS and PDS possibly could be enhanced when they are cotreated with various kinds of known tumor necrosis factor- (TNF-) *α* antagonists [119].

As is mentioned above, PPD could also be an adjuvant agent to achieve more effective anticancer activities. It has been assessed by calcein AM efflux assay that PPD was able to inhibit P-glycoprotein (P-gp) activity as potently as verapamil on MDR cells, while it did not affect ATPase activity of P-gp [77]. Combinations of PPD and docetaxel yield more additive or synergistic activity on established PC-3 tumors compared to animals treated with docetaxel alone [117]. Besides, PPD synergistically enhances cytotoxicity of tamoxifen and mitoxantrone in an estrogen receptor-independent fashion, probably by downregulating Akt activity [21, 51].

As shown in Table 1, PDS including Rc, Rd, Rb1, Rh2, and Rb3 show synergistic activity with chemotherapeutic drugs. Choi et al. [199] demonstrated that PTS isolated from ginseng also has a chemosensitizing effect on P-gp-mediated multidrug resistance (MDR) cells by increasing the intracellular accumulation of drugs through direct interaction with P-gp at the azidopine site. Kitagawa et al. [200] examined that PPT increased the accumulation of P-gp substrate daunorubicin 3.6-fold, more potent than that of CK. Collectively, ginseng types or ginsenosides administration might render an improved efficiency and an ameliorated toxicity of chemotherapy during cancer treatment.

## 4. Conclusion

Observations published in the last years suggest that ginsenoside could be an anticancer agent for various cancers, and the anticancer property of ginsenoside is associated with the induction of apoptosis or autophagy and inhibition of cell proliferation, metastasis, and angiogenesis, as well as modulating the immune system. As the major active components of ginseng types, PTS and PDS ginsenosides have shown wide anticancer properties with respective characteristics. Compared with PTS, PDS ginsenosides (e.g., Rg3) and its metabolites or derivates have stronger therapeutic potential for inhibiting the growth, angiogenesis, metastasis, inflammation, and immune evasion of cancer. On the other hand, PTS and PPT regulate abnormal tumor anabolism, metabolism, and glycolysis in cancer. PTS and its derivatives also depress carcinogenesis and improve the antitumor activity of chemotherapeutic drugs.

As a result of the multiple targets and signaling pathways of ginsenosides, we still could not get a clear understanding of the anticancer effect of ginseng types. But the current research has confirmed the anticancer effect of ginseng types in the aspects mentioned above. Although the research progress on ginseng has greatly promoted its application, how PTS and PDS target cancer-related signaling pathways remains unclear, and the further details and mechanism are still unknown. Thus, it is of importance to understand the characteristics and possible mechanisms associated with the anticancer effects of ginseng derivatives.

## Figures and Tables

**Figure 1:** Major metabolic processes of (a) 20(*S*)-protopanaxadiol- and (b) 20(*S*)-protopanaxatriol-type saponins. CK: compound K, PPD: 20(*S*)-protopanaxadiol, and PPT: 20(*S*)-protopanaxatriol.

**Figure 2:** Therapeutic targets of ginsenosides on cancer. PTS: 20(*S*)-protopanaxadiol saponins, PDS: 20(*S*)-protopanaxatriol saponins, PPT: protopanaxatriol, PPD: protopanaxadiol, and CK: compound K.

**Table 1:** Summary of the anticancer activities of PPD and PDS.

Compounds	Activities	Mechanisms
Protopanaxadiol (PPD)	Antiproliferation	G_1_ phase arrest; promotes melanin production and increases DNA binding sites on the cell surface and cell adhesiveness [69]; stimulates differentiation [31]; induces caspase-dependent apoptosis [70]; activates NF-*κ*B signaling [71]; downregulates PI3K/Akt signaling pathway [50]
	Inhibit tumor growth	Suppresses NF-*κ*B, JNK, and MAPK/ERK signaling pathways [48]; downregulates full-length AR expression and activity and its constitutively active splice variants [6]
	Antimetastasis	Downregulates MMP-9 [72] and MMP-2 [73]
	Antiangiogenesis	Inhibits the proliferation HUVECs
	Synergy and attenuation	Synergies with cyclophosphamide, mitoxantrone, 5-FU, docetaxel, epicatechin, paclitaxel or vinblastine, irinotecan, tamoxifen, or doxorubicin [74–76]. Reverses MDR and inhibits P-gp [77]

Ginsenoside Rg3	Antiproliferation	Induces calcium-dependent apoptosis and autophagy [78]; induces DNA double-strand breaks [79]; downregulates HIF-1*α* expression under hypoxia conditions [80]; downregulates PI3K/Akt [81] and three modules of MAP kinases [82]; inhibits COX-2, NF-*κ*B, phosphorylation of STAT3, ERK1/2, and JNK [83]
	Active tumor suppressors	Induces senescence-like growth arrest by regulating Akt and p53/p21-dependent signaling pathways [61]
	Inhibit cellular metabolism	Increases the cellular GSH/GSSG ratio, enhances the *γ*-GCS activity, and suppresses ROS generation [84]
	Antiangiogenesis	Degrades serum IGF-1 level [85]; downregulates KDR and VEGF expressions [86]; decreases intratumoral microvessel density [87]; inhibits VEGF dependent p38/ERK signaling *in vitro* and inhibits the mobilization of endothelial progenitor cells from the bone marrow microenvironment to the peripheral circulation [88]
	Inhibit tumor growth	Downregulates Wnt/*β*-catenin signaling [54]; decreases HDAC3 and increases acetylation of p53 [63]; decreases FUT4/LeY expression and inhibits the activation of EGFR/MAPK pathway [89]
	Antimetastasis	Suppresses invasion and MMP-9 expression level [90]; inhibits micro-lymphatic metastasis of colorectal neoplasms [91]; blocks hypoxia-induced EMT, activates the ubiquitin-proteasome pathway to promote HIF-1*α* degradation, upregulates E-cadherin via transcriptional suppression of Snail, and downregulates vimentin under hypoxic conditions [92]
	Synergy and attenuation	Reverses P-gp-mediated MDR [93]; increases radiosensitivity [94]; synergies with 5-FU, As_2_O_3_ (arsenic trioxide), capecitabine, cisplatin, CTX, docetaxel, doxorubicin, gemcitabine, gemcitabine plus cisplatin, mitomycin C and tegafur, paclitaxel, ribonuclease inhibitor, suramin, tamoxifen, TRAIL, verapamil, and vinorelbine+cisplatin [95–100]
	Immunomodulation	Improves cellular immunity and stimulates ConA-induced lymphocyte proliferation and augmentation of Th1-type cytokines IL-2 and IFN-*γ* levels in mice [101]; improves the immune function [102]
	Prevent tumorigenesis	Reduces tumor incidence in N:GP(S) newborn mice injected with benzo(a)pyrene [103]; downregulates NF-*κ*B and AP-1 [104]

Ginsenoside Rh2	Antiproliferation	G_1_ phase arrest [105]; induces cell differentiation and reduces telomerase activity [106]; induces Ca^2+^-dependent mitochondrial apoptosis pathway [107]; induces autophagy [78]; activates NF-*κ*B signaling pathway and upregulates TNF-*α* [108]; reduces Akt/mTOR signaling [109]
	Active tumor suppressors	Increases the expression level of DR4 death receptor [65]; upregulates miRNA-128 expression [110]; activates p53 [64]
	Inhibit cellular metabolism	Induces AMPK and p38 MAPK activation. AMPK determines apoptotic sensitivity of cancer cells to Rh2 [111]
	Inhibit tumor growth	Inhibits EGFR signaling through PI3K/Akt/mTOR signaling pathways [112] and upregulation of miR-491 [113]; augment of TGF-*β* receptor signaling [114]
	Antiangiogenesis	Inhibits angiogenesis and lymphangiogenesis and downregulates JAM expression [115]
	Synergy and attenuation	Synergies with cisplatin, betulinic acid, CTX, daunomycin, vinblastine, docetaxel, paclitaxel, and mitoxantrone [116, 117]; reverses P-gp-mediated MDR [118]
	Prevent tumorigenesis	Decreases the tumor incidence in N:GP(S) newborn mice injected with benzo(a)pyrene model [103, 119]

CK/IH-901/M1	Antiproliferation	G_1_ phase arrest [120]. Inhibits telomerase activity and downregulates the human TERT gene [121]; induces mitochondria-dependent apoptotic pathway [122]; inhibits FGFR3 expression and signaling [52]; induces autophagy [123]
	Active tumor suppressors	Inhibits DNA methyltransferase 1 and reactivates epigenetically silenced genes. IC_50_: 20 ± 1.0 *μ*g/mL [124]; upregulates cytochrome C, p53, and Bax expression [125]
	Inhibit cellular metabolism	CAMK-IV/AMPK pathways [126]; inhibits histone deacetylase activity [127]; modulates AMPK-COX-2 signaling [40]
	Anti-inflammation	Inhibits colonic inflammation and tumorigenesis promoted by Western diet. Inhibits tumor xenograft growth. Reduces EGFR and ErbB2 activation and Cox-2 expression [128]
	Inhibit tumor growth	Bid-mediated mitochondrial pathway [42]; increases Ca^2+^ influx, mainly through TRPC channels and by targeting AMPK [129]
	Antimetastasis	Inhibits adhesion, invasion, and spontaneous metastatic growth. Inhibition of AP-1 and MAPK pathways [130]; suppresses the activation of the NF-*κ*B pathway and inhibition of MMP-2/MMP-9 expression [131]
	Antiangiogenesis	Regulates MMP expression, as well as the activity of sphingosine kinase-1 and its related sphingolipid metabolites [132]; blockades of type IV collagenase secretion [133]
	Synergy and attenuation	Synergies with cisplatin, CTX [134]; increases radiosensitivity [135]; decreases the toxicity of irinotecan [136]
	Prevent tumorigenesis	Prevents tumorigenesis of aberrant crypts in C57BL:6 mice colonized with ginseng-hydrolyzing bacteria

Ginsenoside Rb1	Antiproliferation	Increases the expression levels of caspase-3 and caspase-8 [137]
	Antiangiogenesis	Inhibits the HGF/SF-induced chemoinvasion. Inhibits tyrosine kinase [10]; regulates pigment epithelium-derived factor through the estrogen *β* receptor [138]
	Attenuation	Reduces CTX-induced DNA damage and apoptosis effects [139]
	Chemoprevention	Induces cytochrome P450 1A1 expression. Aryl hydrocarbon receptor [140]

Ginsenoside Rb2	Antiproliferation	Increases the expression levels of caspase-3 and caspase-8 [137]
	Antimetastasis	Inhibits the adhesion and invasion and suppression of MMP-2 [141]
	Prevent tumorigenesis	Prevents the downregulation of gap junctional intercellular communication by TPA and hydrogen peroxide [142]

Ginsenoside Rb3	Antiproliferation	Inhibits DNA transferring and duplication [143]; inhibits RNF-*α*-induced NF-*κ*B activity and inhibits COX-2 and iNOS mRNA levels [144]
	Synergy and attenuation	Increases cisplatin's antiproliferative activity in MCF-7 cells [145]

Ginsenoside Rc	Antiproliferation	Antiproliferation of HCT-116 and HT-29 cells [146]
	Synergy and attenuation	Reverses MDR, reduces the activity of the efflux pump, enhances T cell proliferation, and increases the NK cell activity [147]

Ginsenoside Rd	Antiproliferation	Inhibits the chymotrypsin-like activity of 26S proteasome [148]; induces apoptosis and reduces oxidative stress and associates with DNA replication and repair, protein synthesis and degradation, mutagenesis, and metastasis [149]
	Antimetastasis	Blocks MMP activation and MAPK signaling pathways [55]
	Synergy and attenuation	Reverses MDR, reduces the activity of the efflux pump, enhances T cell proliferation, and increases the NK cell activity [147]

Ginsenoside Rk1	Antiproliferation	Induces apoptosis, upregulation of Fas, FasL, and Bax, and downregulation of procaspase-8 and procaspase-3, mutant p53, and Bcl-2 [59]

Ginsenoside Rs3	Antiproliferation	G_1_/S phase arrest. Elevates protein levels of p53 and p21^WAF1^ and downregulates the activities of the cyclin-dependent kinases [60]

Ginsenoside F2	Antiproliferation	Induces apoptosis accompanied by protective autophagy. Activates intrinsic apoptotic pathway and mitochondrial dysfunction [150]
	Inhibit tumor growth	IC_50_: 49.9 ± 4.2 *μ*M. Accumulation of ROS and activating the ASK-1/JNK signaling pathway [19]
	Antimetastasis	IC_50_: 50 *μ*g/mL. Activation of caspase-3 and caspase-8 and inhibition of MMP-9 [151]

Ginsenosides Mb, Mc, and Mx	Antiproliferation	Antiproliferation of HCT-116 and HT-29 cells [146], as well as HL-60, HGC-27, Colon205, and Du145 cells [152]

**Table 2:** Summary of the anticancer activities of PPT and PTS.

Effects	Activities	Mechanisms
Ginsenosides F1 and F5	Antiproliferation	Induces chromatin condensation and increases sub-G_1_hypodiploid cells. IC_50_: 23.2 *μ*M and 62.4 *μ*M [153]

Ginsenoside Re	Antiproliferation	Increases GSH/GSSG ratio, enhances the *γ*-GCS activity, and suppresses ROS generation [84]; inhibits the transferring and duplication of DNA [143]
	Synergy and attenuation	Synergies with cisplatin. Increases cisplatin's antiproliferative activity [145]

Ginsenoside Rf	Antiproliferation	G_2_/M phase arrest. IC_50_: 11.36 *μ*M. Upregulates Bax and downregulates Bcl-2, CDK1, and cyclin B1, activates caspase-3 and caspase-9, and releases cytochrome C [154]

Ginsenoside Rg1	Antiproliferation	Inhibits ubiquitin activating enzyme (E_1_) activity [155]; S phase arrest and induces cell senescence [156]; increases the expression levels of caspase-3 and caspase-8; induces apoptosis [137]; inhibits EpoR-mediated JAK2/STAT5 signal pathway [157]
	Immunomodulation	Activates tumor killer cells and enhances the production of NO from IFN-*γ* activated-macrophages [158]
	Inhibit tumor growth	Inhibits colon cancer growth. Downregulates the expression of cyclin D1, PCNA, and VEGF [159]
	Antimetastasis	Suppresses TPA-induced tumor cell invasion and migration by inhibition of NF-*κ*B-dependent MMP-9 expression [160]; inhibits transforming growth factor-*β*1-induced epithelial-to-mesenchymal transition [161]
	Synergy and attenuation	Synergist with IL-2. Activates lymphokine activated killer cells as a synergistic of IL-2 [162]
	Chemoprevention	Induces cytochrome P450 1A1 expression. Aryl hydrocarbon receptor [140]

Ginsenoside Rg2	Antiproliferation	IC_50_: 9.0 *μ*M [153]

Ginsenoside Rh1	Antiproliferation	Induces differentiation. Stimulates the nuclear translocation of glucocorticoid receptor [163]; induces apoptosis [30]
	Antimetastasis	Inhibits the invasion and migration. Suppresses MMP-1 expression through inhibition of AP-1 and MAPK signaling pathway [164]; inhibits MMPs gene expression by suppressing MAPKs, PI3K/Akt, and downstream NF-*κ*B and AP-1 [165]

Notoginsenoside R1	Antiproliferation	Induces differentiation; affects synthesis of DNA and RNA [166]; upregulates p53 gene and downregulates Bcl-2 gene [167]

Protopanaxatriol (PPT)	Antiproliferation	Increases sub-G_1_ cells [168]; induces apoptosis. Activation of p53 and p21 and downregulation of CDK2, cyclin E and cyclin D1, and PCNA [58]
	Antiangiogenesis	Inhibits the proliferative activity of HUVECs in a dose-dependent manner. EC_50_: 6.64 *μ*g/mL [67]
	Antimetastasis	Enhances natural-killer cytotoxicity by esterified protopanaxatriol [169]; inhibits invasion and downregulation of MMP-9 [72]
	Synergy and attenuation	Reverses daunomycin and vinblastine resistance [170]; synergies with mitoxantrone; inhibits BCRP-associated vanadate sensitive ATPase activity [21]

## Abbreviations

25-OCH3-PPD: 20(*S*)-25-Methoxyl-dammarane-3*β*,12*β*,20-triol
25-OH-PPD: 20(*R*)-Dammarane-3*β*,12*β*,20,25-tetrol
Akt: Protein kinase B
ALL: Acute lymphoblastic leukemia
AMPK: AMP-activated protein kinase
cAMP: Cyclic AMP
AP-1: Activator protein-1
AR: Androgen receptor
ASK-1: Apoptosis signal regulating kinase-1
ATP: Adenosine triphosphate
Bcl-2: B-cell lymphoma-2
BCRP: Breast cancer resistance protein
CDK: Cyclin-dependent kinase
CK: Compound K
COX-2: Cyclooxygenase-2
CTX: Cyclophosphamide
DC: Dendritic cell
EGFR: Epidermal growth factor receptor
EMT: Epithelial-mesenchymal transition
ERK: Extracellular signal-regulated kinase
bFGF: Basic fibroblast growth factor
FGFR3: Fibroblast growth factor receptor 3
FUT4: Fucosyltransferase 4
GCS: Glasgow Coma Scale
GR: Glucocorticoid receptor
GSH: Glutathione
GSSG: Oxidized glutathione
HDAC3: Histone deacetylase 3
HGF/SF: Hepatocyte growth factor/scatter factor
HIF-1: Hypoxia inducible factor-1
HUVEC: Human umbilical vein endothelial cell
IFN: Interferon
IL: Interleukin
JAK: Janus activated kinase
JAM: Junctional adhesion molecule
JNK: c-Jun N-terminal kinase
KDR: Kinase insert domain receptor
MAPK: Mitogen-activated protein kinase
MDR: Multidrug resistance
MMP: Matrix metalloproteinase
MVD: Mevalonate (diphosphate) decarboxylase
NADPH: Nicotinamide adenine dinucleotide phosphate
NF-*κ*B: Nuclear factor-kappa B
NO: Nitric oxide
NQO1: NADPH quinone oxidoreductase 1
OCK: 3-O-Oleoyl compound K
PARP: Poly(ADP-ribose) polymerase
PCNA: Proliferating cell nuclear antigen
PDS: 20(*S*)-Protopanaxadiol saponin
PGE_2_: Prostaglandin E_2_
PI3K: Phosphatidylinositol 3-kinase
PPD: 20(*S*)-Protopanaxadiol
PPT: 20(*S*)-Protopanaxatriol
PTEN: Phosphatase and tensin homolog
PTS: 20(*S*)-Protopanaxatriol saponin
RNF-*α*: RING finger protein-alpha
ROS: Reactive oxygen species
TERT: Telomerase reverse transcriptase
TGF: Transforming growth factor
TPA: 12-O-Tetradecanoylphorbol-13-acetate
TRAIL: Tumor necrosis factor-related apoptosis-inducing ligand
TRPC: Transient receptor potential channel
VEGF: Vascular endothelial growth factor.
